The article "A Cost Allocation Decision Model for Air Pollution Control" was retracted in 2023. Reasons: unreliable results or conclusions; concerns about the data; concerns about the peer review; concerns about the citations.

# A Cost Allocation Decision Model for Air Pollution Control

**DOI:** 10.1155/2022/4116527

**Published:** 2022-01-31

**Authors:** Dong-Sheng Qin, Chang-Yuan Gao

**Affiliations:** Harbin University of Science and Technology, Harbin, China

## Abstract

Air pollution control as the background of a cost allocation method is based on the Shapley value to determine the core stakeholder, so fair pollution control projects and the establishment of the atmospheric pollution of governance cost allocation model are put forward for the solution of air pollution coordinated by the government supervision and the atmospheric pollution control collaborative group. The results show that the cost allocation model of air pollution control based on Shapley value is more reasonable, and the cost of stakeholders is reduced to a certain extent, and the risk of the participants is reduced so that it maximizes social benefits.

## 1. Introduction

Over the past 30 years of the Reform and Opening-up policy, China has made some progress in air pollution prevention and control. A part of single atmospheric pollutants has reached the emission standard step by step. However, new pollution caused by the mixing of multiple pollution sources has attracted widespread attention with the complexity of production and living activities. PM2.5 or haze is formed by a mixed reaction of various pollutants, such as gases and particulates, including volatile organic compounds (VOCs). Exposure to fine particulate matter (PM2.5) with a diameter of < 2.5 μm is a recognized cause of respiratory diseases in children [1]. At present, the generation of air pollutants is continuing to increase. Effective pollution prevention and control should decrease the increment and storage of pollutants. At present, the problem of air pollution control is still facing many difficulties and needs to be solved urgently.

In my country's urban development system, the urban development of the Beijing-Tianjin-Hebei region has driven the overall economic development of our country, but the environmental problems in these areas have gradually become the main concern of people. [2] The Beijing-Tianjin-Hebei region, which is a key area of pollution prevention and control, suffers from grave ecological and environmental problems, especially serious air pollution and frequent haze. At the same time, the Beijing-Tianjin-Hebei region, which has a resource-dependent economy dominated by clusters of heavy industries, has long borne the highest PM2.5 pollution levels in China, prompting serious concerns about the region's disease burden. [3] The overall air quality in the Beijing-Tianjin-Hebei region affects each other and cannot be prevented and controlled individually. It is urgent to strengthen regional ecological protection and construction. However, the integration of the Beijing-Tianjin-Hebei region is still at an early stage, and many systems need to be further established and refined. It is also difficult to significantly improve the quality of the atmospheric environment in the short term. Under this circumstance, coordinating the contradiction between the environmental demand and environmental capacity of the Beijing-Tianjin-Hebei region is prominent.

Noncooperative policies for transboundary pollution abatement are inefficient and ineffective, but cooperative policies for pollution abatement are seldom successful in regions that have different development goals and conflicting interests. [4] To reduce the harm of haze to the life and health of residents and accelerate the coordinated prevention and control of air pollution in the Beijing-Tianjin-Hebei region require more resources and capital investment. However, the Beijing-Tianjin-Hebei cooperation has not clearly defined and divided rights, responsibilities, and benefits in air pollution prevention and control, especially the cost-sharing mechanism, so it is difficult to achieve effective integration.

In response to the above problems, this paper conducts a theoretical analysis on the cost allocation of the Beijing-Tianjin-Hebei cooperation in air pollution control. We propose to establish a cost-sharing model of atmospheric pollution in Beijing, Tianjin, and Hebei by using Shapley value. This model can better identify stakeholders in the cooperative governance, maximize the overall and individual interests, reduce the cost of air pollution prevention and control, and finally solve the coordination problem of air pollution control in Beijing, Tianjin, and Hebei.

## 2. Literature Review

Haze pollution not only negatively influences public health but also causes great economic losses [5, 6]. In the existing research on air pollution control, the main focus is on the causes of air pollution and the control measures of air pollution. Yang et al. quantitatively evaluated the vulnerability of the atmospheric environment in the Beijing-Tianjin-Hebei region through space-time comparison [7]. The relationship between atmospheric environmental vulnerability and exposure index, sensitivity index, and adaptability index is helpful to analyze atmospheric environmental vulnerability. The results show that the air environment vulnerability of 13 cities in the Beijing-Tianjin-Hebei region shows obvious spatial heterogeneity. Liang and Wang systematically summarized the Beijing-Tianjin-Hebei urban agglomeration implemented air pollution control mode, which is multilevel, cross regional, and multidirectional [8]. This includes a state-agglomeration-city linkage structure, multiprovincial, and cross-regional linkage governance, and multidirectional linkage mechanisms involving industrial access, energy structure, green transportation, cross-regional assistance, monitoring and early warning, consultation, and accountability to analyze the temporal and spatial characteristics by using the concentration data of six kinds of air pollutants. Sun et al. selected indicators from the three aspects of air pollution characteristics, natural condition characteristics, and trade characteristics, and used the entropy-top SIS method to determine the priority order of the JPCAP region [9]. By determining the key areas of four regions, key areas of air pollution control were identified, providing practical guidance and theoretical basis for regional joint control of air pollution. Piersanti et al. discussed the scenarios developed for 2030 in Italy's National Air Pollution Control Programme, using 2010 as the reference year, and also used these scenarios to provide a comprehensive approach to calculating the impact of the plan on health effects (mortality) and associated costs, providing an important framework and assessing measures to reduce air pollution with an integrated approach [10]. Ikeuchi et al. proposed that health risks caused by PM2.5 would increase with the decrease of precipitation duration and incidence [11]. Schwartz et al. believed that particulate air pollution at common concentrations is associated with daily death [12]. Gulia et al. highlighted the problem of high spatiotemporal variation of air pollution levels in urban areas and the methods that can be used to eliminate pollutants. The efficiency of the prototypes/devices developed using these processes has also been compared worldwide, and studies have shown that such controls would be very useful in reducing air pollution in hot spots with large spatiotemporal variability [13].

Given the formation reasons of haze and its harm to human health, Elżbieta believed that the biggest cause of smog and air pollution is the burning of garbage in the stoves; other causes include exhaust from large factories, burning coal in the stoves, and automobile exhaust [14]. Urbanization, industrialization, and increasing fossil fuel consumption are generally identified as the main contributors to poor air quality [15]. Zhao and Yuan innovatively used precipitation as an instrumental variable to alleviate the endogeneity of haze pollution variable and found that haze pollution seriously reduces the quality of China's economic development. The loss of labor supply, deurbanization, and interruption of human capital are the three transmission channels through which haze pollution affects the quality of China's economic development [16]. Wang et al. studied the changes in the physical and chemical properties of air particles collected in Beijing during the typical transition from haze to dust [17]. The study found that detailed information on the physical and chemical properties of atmospheric particles in the typical heavy pollution process could be provided in a short time, and such short-term changes should be taken into account to more accurately assess the environmental, climatic, and health impacts of airborne particulate matter. Intense economic and human activities in megacities lead to air pollution emissions, resulting in high concentrations of air pollutants in the atmosphere that harm human health, cause regional haze and acid deposition, damage crops, affect regional air quality, and contribute to climate change [18]. Zhang et al. studied the diurnal variation of atmospheric boundary layer height, analyzed temperature, wind direction and vertical structure of wind, and characteristics of velocity in the boundary layer; the weak vertical exchange between the boundary layer and the upper layer will promote the formation of fog and haze [19].

SOx, NOx, COx, volatile organic compounds (VOCs), and Hg vapor directly and indirectly harm the atmospheric environment and human health by contributing to the formation of photochemical smog, acid rain, and haze and posing risks of potential toxicity (e.g., carcinogenicity) [20]. Wang and Yuan tested the impact of air pollution control on ecological total factor energy efficiency and the moderating effect of ownership structure by using panel data of 37 subindustries of China's industrial sectors from 2003 to 2014. They found that high-pollution industries had a significant short-term positive impact, while medium-pollution industries had a significant short-term negative impact. Low pollution industries have a significant long-term negative impact. Finally, some concrete policy suggestions are put forward [21]. Kim et al. determined the causal relationship between the risk perception of particulate matter and satisfaction of outdoor activities in South Korea, conducted an online survey of 412 people, and conducted confirmatory factor analysis using the structural equation model. The results showed that the perceived risk of particulate matter was higher when people had no interest or trust in public opinion or policy, which increased people's perception of health risks and, in turn, reduced their satisfaction with outdoor activities [22]. Zhao et al. studied the Beijing-Tianjin-Hebei region as an example, used the Shapley value method to reasonably distribute the model benefits, construct the optimal emission reduction plan, and determine the optimal annual decision of each province. The results show that the model reduces the total cost of SO_2_ pollution reduction [23]. Gao et al. evaluated the risk of particulate pollution to human health by comparing samples collected from seven different functional areas in Beijing [24].

At present, haze air pollution seriously harms global human health. Many scholars at home and abroad have made detailed explanations on the sources of air pollutants, mainly from organic compounds such as SOx, NOx, and COx, open incineration of garbage, and automobile exhaust emissions. For the study of air pollution, many scholars focus on empirical research. However, the Shapley value method is a model of the income distribution of participants in dynamic cooperative alliances. At present, the Shapely value method is mainly used to solve the income distribution in cooperative projects at home and abroad. The Shapley value method is seldom used to study the cost of air pollution control.

In this paper, the cost of air pollution control is allocated according to the Shapley value method. Compared with the existing research work, this model avoids equal distribution and other relatively simple distribution to a certain extent, which is scientific, reasonable, and fair. This paper establishes an air pollution control cost-sharing model based on the Shapley value and determines the core stakeholders to make the cost allocation more reasonable, scientific, and fair. The Shapley model reduces the charges of each stakeholder, disperses the risks of participants to a certain extent, and effectively ensures the smooth progress of the project. We found that the cost distribution model based on Shapley value can optimize the cost and maximize the social benefit. Because air pollution control needs a long process, the reduction of cost and risk can effectively ensure the completion of air pollution control, which plays an important role in promoting air pollution control.

## 3. Basic Theory of Air Pollution Control Cost Allocation

### 3.1. Shapley Value Method

Let *I*={1,2,…, *n*} be the total number of project participants, *S* be any subset of *I*, and *V* be the characteristic function defined above *I*, that is, the benefit of a certain cooperation *S*.

(1) $$\begin{array}{c} V\left(\emptyset \right)=0\left(1\right),\\ V\left(S_{1}\cup S_{2}\right)\geq V\left(S_{1}\right)+V\left(S_{2}\right),S_{1}\cap S_{2}=\emptyset . \end{array}$$

With *Y*_*i*_ said I in the case of a project I partners from the alliance profit maximum *V*_(*I*)_ in income, namely, the income gained by the each participant in the I uses letters to represent *Y*, this model is a cost allocation which should not only meet the rationality of overall but also at the same time to meet the individual rationality [25, 26], as shown below:

(2) $$\begin{array}{c} \text{the overall rational }:\;\sum_{i=1}^{n}Y_{i}=V\left(I\right),\;i=1,2,\ldots ,n,\\ \text{individual rationality }:\;Yi\geq V\left(i\right),\;i=1,2,\ldots ,n, \end{array}$$

where *V*(*I*) represents the benefit that I, a participant, can obtain by completing the project alone, and *V*(*I*) represents the maximum benefit that can be obtained in many cooperative alliances [27, 28]. At this point, we get the Shapley value we want to find, which is called *Y*_*i*_ (*v*):

(3) $$\begin{array}{c} Y_{i}\left(V\right)=\sum \sum_{S_{i\in s}}W\left(\left|s\right|\right)\left[V\left(S\right)-V\left(s\backslash i\right)\right],\;i=1,2\ldots n,\\ \;W\left(\left|S\right|\right)=\frac{\left(n-\left|S\right|\right)!\left(\left|S\right|-1\right)!}{n!}, \end{array}$$

where S is a subset of all combinations of *I*, and |*S*| is the number of project-related stakeholders in a collaboration *S*, and *W*(|*S*|) is the weight. *V*(*S*) refers to the cooperation benefits obtained or costs borne by this subset S, and *V*(*S*/*i*) refers to the benefits obtained or costs borne by other members of S after the elimination of participant I [29].

### 3.2. Stakeholder Theory

Rowley, a foreign scholar, was the first to establish the stakeholder theory. In a narrow sense, a stakeholder means that an individual and a group participate in the same project, provide human, financial, and other resources in the project, bear a part of the project risks, and finally share interests [30, 31]. In the late 1990s, there emerged a method represented by Mitchell and Wood, called the “Mitchell scoring method,” which mainly divided legitimacy, power, and urgency into three attributes. According to these three attributes, stakeholders can be divided into three types: the first type is the defining stakeholder, which has three attributes at the same time and is the primary object to be paid attention to. The second type is the anticipatory stakeholder, with any combination of two attributes. The third type is the potential stakeholder, in which participants have only one of the three characteristics [32].

## 4. Air Pollution Control Cost Allocation Model

### 4.1. Core Stakeholders of Air Pollution Control Cost Allocation Project

According to the participation of each participant in the process of air pollution control project and the degree of influence of each participant on air pollution control, [33] stakeholders in the air pollution control model are divided into three categories through analysis, as shown in Table 1.

In atmospheric pollution control projects, as core stakeholders are the key members of air pollution control and also the main body to share the cost of air pollution, they play a vital role in air pollution control, so it is particularly important to determine the cost allocation among core stakeholders [34].

### 4.2. Cost Allocation Model of Air Pollution Control Based on Shapley Value

Based on the above analysis of stakeholders, a model is established for the allocation process of air pollution treatment costs. Combined with the relevant knowledge of Shapley value, hypotheses are firstly proposed for the model. The main hypotheses are as follows:

Assume that participants *I* = {1,2, ..., *n*}, including government departments of two places and enterprises of two places, are represented by A,B,C,D,E, and F, respectively. A represents government departments of Beijing, B represents enterprises of Beijing, C represents the government of Hebei, D represents enterprises of Hebei, E represents the government of Tianjin, and F represents enterprises of Tianjin as shown in Table 2.

Based on the analysis of the above characteristic functions and the Shapley value method, the cost allocation model of regional cooperative air pollution control is established, which is mainly calculated according to the following two formulas.

(4) $$\begin{array}{c} W\left(\left|S\right|\right)=\frac{\left(n-\left|s\right|!\right)\left(\left|s\right|-1\right)!}{n!}, \end{array}$$

(5) $$\begin{array}{c} Y_{i}\left(V\right)=\sum_{S_{i}\in S}W\left(\left|S\right|\right)\left[V\left(S\right)-V\left(S/i\right)\right],\;i=1,2,\ldots ,n. \end{array}$$

### 4.3. Cost Allocation of Beijing Government Departments in the Air Pollution Control Project Alliance

The values in the table are calculated according to formula (4) and formula (5). The constituent elements in the subset S represent the stakeholders involved in the project. They, respectively, say that the cooperative alliance V (S) participated by Beijing government departments represents the air pollution control costs borne by the cooperative alliance participated by the Beijing municipal government V (S/I) represents the removal of Beijing city. After the government, this cooperative alliance would have borne the cost and [*V*(*S*) − *V*(*S*/*i*)] refers to the cost borne by the project with the participation of Beijing municipal government minus the cost borne by the project without the participation of Beijing municipal government. W(|S|) refers to the proportion of this cooperation alliance in cooperation with the participation of Beijing municipal government. The sum of W(|S|) is 1. W(|S|)[*V*(*S*) − *V*(*S*/*i*)] represents the Shapley value of Beijing municipal Government in this cooperative alliance, from which we can get the best cost allocation of Beijing municipal government. According to the formula, the final cost that Beijing municipal government should bear is as shown in Table 3.

(6) $$\begin{array}{c} Y_{i}\left(V\right)=\frac{1}{6}\;V\left(S1\right)+\frac{1}{30}\left[V\left(S5\right)-V\left(S2\right)\right]+\frac{1}{30}\left[V\left(S7\right)-V\left(S4\right)\right]+\frac{1}{30}\left[V\left(S9\right)-V\left(S3\right)\right]\\ +\frac{1}{30}\left[V\left(S7\right)-V\left(S4\right)\right]+\frac{1}{30}\left[V\left(S9\right)-V\left(S3\right)\right]\frac{1}{60}\left[V\left(S11\right)-V\left(S6\right)\right]+\frac{1}{60}\left[V\left(S13\right)-V\left(S8\right)\right]\\ +\frac{1}{60}\left[V\left(S14\right)-V\left(S10\right)\right]+\frac{1}{60}\left[V\left(S15\right)-V\left(S12\right)\right]+\frac{1}{30}\left[V\left(S19\right)-\;V\left(S17\right)\right]+\frac{1}{30}\left[V\left(S23\right)-V\left(S16\right)\right]\\ +\frac{1}{60}\left[V\left(S31\right)-V\left(S21\right)\right]+\frac{1}{60}\left[V\left(S32\right)-\;V\left(S20\right)\right]+\frac{1}{60}\left[V\left(S33\right)-V\left(S18\right)\right]+\frac{1}{60}\left[V\left(S35\right)-V\left(S24\right)\right]\\ +\frac{1}{60}\left[V\left(S37\right)-V\left(S26\right)\right]+\frac{1}{60}\left[V\left(S38\right)-V\left(S22\right)\right]+\frac{1}{60}\left[V\left(S40\right)-V\left(S25\right)\right]+\frac{1}{60}\left[V\left(S43\right)-V\left(S34\right)\right]\\ +\frac{1}{60}\left[V\left(S45\right)-V\left(S36\right)\right]+\frac{1}{60}\left[V\left(S49\right)-V\left(S39\right)\right]\frac{1}{60}\left[V\left(S50\right)-V\left(S27\right)\right]+\frac{1}{60}\left[V\left(S51\right)-V\left(S29\right)\right]\\ +\frac{1}{60}\left[V\left(S52\right)-V\left(S41\right)\right]+\frac{1}{60}\left[V\left(S53\right)-V\left(S28\right)\right]+\frac{1}{60}\left[V\left(S54\right)-V\left(S42\right)\right]+\frac{1}{60}\left[V\left(S55\right)-V\left(S30\right)\right]\\ +\frac{1}{30}\left[V\left(S58\right)-V\left(S44\right)\right]+\frac{1}{30}\left[V\left(S59\right)-V\left(S48\right)\right]+\frac{1}{30}\left[V\left(S60\right)-V\left(S46\right)\right]+\frac{1}{30}\left[V\left(S61\right)-V\left(S47\right)\right]\\ +\frac{1}{30}\left[V\left(S62\right)-\;V\left(S56\right)\right]+\frac{1}{6}\left[V\left(S63\right)-\;V\left(S57\right)\right]. \end{array}$$

According to the formula, the final cost that Beijing enterprises should bear is

(7) $$\begin{array}{c} Y_{i}\left(V\right)=\frac{1}{6}V\left(S2\right)+\frac{1}{30}\left[V\left(S5\right)-V\left(S1\right)\right]+\frac{1}{30}\left[V\left(S10\right)-V\left(S4\right)\right]+\frac{1}{60}\left[V\left(S12\right)-V\left(S6\right)\right]+\frac{1}{60}\left[V\left(S13\right)-\;V\left(S9\right)\right]+\frac{1}{60}\left[V\left(S14\right)-\;V\left(S7\right)\right]\\ +\frac{1}{60}\left[V\left(S15\right)-\;V\left(S11\right)\right]+\frac{1}{30}\left[V\left(S20\right)-\;V\left(S17\right)\right]+\frac{1}{30}\left[V\left(S20\right)-V\left(S17\right)\right]+\frac{1}{30}\left[V\left(S22\right)-V\left(S16\right)\right]+\frac{1}{60}\left[V\left(S31\right)-V\left(S5\right)\right]\\ +\frac{1}{60}\left[V\left(S32\right)-V\left(S19\right)\right]+\frac{1}{60}\left[V\left(S34\right)-V\left(S18\right)\right]+\frac{1}{60}\left[V\left(S36\right)-V\left(S25\right)\right]+\frac{1}{60}\left[V\left(S39\right)-V\left(S24\right)\right]+\frac{1}{60}\left[V\left(S41\right)-V\left(S26\right)\right]\\ +\frac{1}{60}\left[V\left(S42\right)-V\left(S22\right)\right]+\frac{1}{60}\left[V\left(S43\right)-V\left(S33\right)\right]+\frac{1}{60}\left[V\left(S45\right)-V\left(S40\right)\right]+\frac{1}{60}\left[V\left(S46\right)-V\left(S29\right)\right]+\frac{1}{60}\left[V\left(S47\right)-V\left(S28\right)\right]\\ +\frac{1}{60}\left[V\left(S48\right)-V\left(S30\right)\right]+\frac{1}{60}\left[V\left(S49\right)-V\left(S35\right)\right]+\frac{1}{60}\left[V\left(S52\right)-V\left(S-37\right)\right]+\frac{1}{60}\left[V\left(S54\right)-V\left(S38\right)\right]+\frac{1}{60}\left[V\left(S56\right)-V\left(S27\right)\right]\\ +\frac{1}{30}\left[V\left(S57\right)-V\left(S44\right)\right]+\frac{1}{30}\left[V\left(S59\right)-V\left(S55\right)\right]+\frac{1}{30}\left[V\left(S60\right)-V\left(S51\right)\right]+\frac{1}{30}\left[V\left(S61\right)-V\left(S53\right)\right]+\frac{1}{30}\left[V\left(S62\right)-\;V\left(S50\right)\right]\\ +\frac{1}{6}\;\left[V\left(S63\right)-\;V\left(S58\right)\right]. \end{array}$$

According to the formula, the final cost that Hebei government should bear is

(8) $$\begin{array}{c} Y_{i}\left(V\right)=\frac{1}{6}V\left(S3\right)+\frac{1}{30}\left[V\left(S6\right)-V\left(S4\right)\right]+\frac{1}{30}\left[V\left(S8\right)-V\left(S2\right)\right]+\frac{1}{30}\left[V\left(S9\right)-V\left(S1\right)\right]+\frac{1}{60}\left[V\left(S11\right)-\;V\left(S7\right)\right]+\frac{1}{60}\left[V\left(S12\right)-\;V\left(S8\right)\right]\\ +\frac{1}{60}\left[V\left(S13\right)-\;V\left(S5\right)\right]+\frac{1}{60}\left[V\left(S15\right)-\;V\left(S14\right)\right]+\frac{1}{30}\left[V\left(S20\right)-V\left(S17\right)\right]+\frac{1}{30}\left[V\left(S24\right)-V\left(S16\right)\right]+\frac{1}{60}\left[V\left(S26\right)-V\left(S17\right)\right]\\ +\frac{1}{60}\left[V\left(S27\right)-V\left(S22\right)\right]+\frac{1}{60}\left[V\left(S28\right)-V\left(S25\right)\right]+\frac{1}{60}\left[V\left(S29\right)-V\left(S18\right)\right]+\frac{1}{60}\left[V\left(S35\right)-V\left(S25\right)\right]+\frac{1}{60}\left[V\left(S37\right)-V\left(S19\right)\right]\\ +\frac{1}{60}\left[V\left(S39\right)-V\left(S21\right)\right]+\frac{1}{60}\left[V\left(S41\right)-V\left(S20\right)\right]+\frac{1}{60}\left[V\left(S44\right)-V\left(S30\right)\right]+\frac{1}{60}\left[V\left(S46\right)-V\left(S34\right)\right]+\frac{1}{60}\left[V\left(S47\right)-V\left(S36\right)\right]\\ +\frac{1}{60}\left[V\left(S49\right)-V\left(S31\right)\right]+\frac{1}{60}\left[V\left(S50\right)-V\left(S38\right)\right]+\frac{1}{60}\left[V\left(S51\right)-V\left(S-33\right)\right]+\frac{1}{60}\left[V\left(S52\right)-V\left(S32\right)\right]+\frac{1}{60}\left[V\left(S53\right)-V\left(S27\right)\right]\\ +\frac{1}{30}\left[V\left(S56\right)-V\left(S44\right)\right]+\frac{1}{30}\left[V\left(S57\right)-V\left(S40\right)\right]+\frac{1}{30}\left[V\left(S58\right)-V\left(S55\right)\right]+\frac{1}{30}\left[V\left(S60\right)-V\left(S43\right)\right]+\frac{1}{30}\left[V\left(S62\right)-\;V\left(S45\right)\right]\\ +\frac{1}{6}\;\left[V\left(S63\right)-\;V\left(S59\right)\right]. \end{array}$$

According to the formula, the final cost that Hebei enterprises should bear is

(9) $$\begin{array}{c} Y_{i}\;\left(V\right)=\frac{1}{6}V\left(S4\right)+\frac{1}{30}\left[V\left(S6\right)-V\left(S3\right)\right]+\frac{1}{30}\left[V\left(S7\right)-V\left(S1\right)\right]+\frac{1}{30}\left[V\left(S10\right)-V\left(S2\right)\right]+\frac{1}{60}\left[V\left(S11\right)-V\left(S9\right)\right]\\ +\frac{1}{60}\left[V\left(S12\right)-V\left(S8\right)\right]+\frac{1}{60}\left[V\left(S14\right)-V\left(S5\right)\right]+\frac{1}{60}\left[V\left(S15\right)-V\left(S13\right)\right]+\frac{1}{30}\left[V\left(S22\right)-V\left(S16\right)\right]\\ +\frac{1}{30}\left[V\left(S26\right)-V\left(S14\right)\right]+\frac{1}{60}\left[V\left(S27\right)-V\left(S26\right)\right]+\frac{1}{60}\left.\left[V\left(S29\right)-V\left(S18\right)\right]\right]+\frac{1}{60}\left[V\left(S35\right)-V\left(S20\right)\right]\\ +\frac{1}{60}\left[V\left(S37\right)-V\left(S23\right)\right]+\frac{1}{60}\left[V\left(S39\right)-V\left(S19\right)\right]+\frac{1}{60}\left[V\left(S41\right)-V\left(S21\right)\right]+\frac{1}{60}\left[V\left(S43\right)-V\left(S29\right)\right]\\ +\frac{1}{60}\left[V\left(S44\right)-V\left(S32\right)\right]+\frac{1}{60}\left[V\left(S46\right)-V\left(S41\right)\right]+\frac{1}{60}\left[V\left(S47\right)-V\left(S34\right)\right]+\frac{1}{60}\left[V\left(S49\right)-V\left(S35\right)\right]\\ +\frac{1}{60}\left[V\left(S52\right)-V\left(S37\right)\right]+\frac{1}{60}\left[V\left(S53\right)-V\left(S31\right)\right]+\frac{1}{60}\left[V\left(S54\right)-V\left(S33\right)\right]+\frac{1}{60}\left[V\left(S55\right)-V\left(S39\right)\right]\\ +\frac{1}{60}\left[V\left(S56\right)-V\left(S46\right)\right]+\frac{1}{30}\left[V\left(S57\right)-V\left(S51\right)\right]+\frac{1}{30}\left[V\left(S58\right)-V\left(S43\right)\right]+\frac{1}{30}\left[V\left(S59\right)-\;V\left(S52\right)\right]\\ +\frac{1}{30}\left[V\left(S61\right)-\;V\left(S49\right)\right]+\frac{1}{30}\left[V\left(S62\right)-\;V\left(S60\right)\right]+\frac{1}{6}\left[V\left(S25\right)-\;V\left(S17\right)\right]. \end{array}$$

According to the formula, the final cost that Tianjin government should bear is

(10) $$\begin{array}{c} Y_{i}\;\left(V\right)=\frac{1}{6}V\left(S16\right)+\frac{1}{30}\left[V\left(S18\right)-V\left(S17\right)\right]+\frac{1}{30}\left[V\left(S21\right)-V\left(S2\right)\right]+\frac{1}{30}\left[V\left(S22\right)-V\left(S3\right)\right]+\frac{1}{30}\left[V\left(S23\right)-V\left(S6\right)\right]\\ +\frac{1}{60}\left[V\left(S24\right)-V\left(S26\right)\right]+\frac{1}{60}\left[V\left(S27\right)-V\left(S25\right)\right]+\frac{1}{60}\left[V\left(S29\right)-V\left(S5\right)\right]+\frac{1}{30}\left[V\left(S30\right)-V\left(S19\right)\right]\\ +\frac{1}{30}\left[V\left(S31\right)-V\left(S20\right)\right]+\frac{1}{60}\left[V\left(S27\right)-V\left(S26\right)\right]+\frac{1}{60}\left.\left[V\left(S39\right)-V\left(S41\right)\right]\right]+\frac{1}{60}\left[V\left(S42\right)-V\left(S28\right)\right]\\ +\frac{1}{60}\left[V\left(S35\right)-V\left(S32\right)\right]+\frac{1}{60}\left[V\left(S38\right)-V\left(S28\right)\right]+\frac{1}{60}\left[V\left(S41\right)-V\left(S21\right)\right]+\frac{1}{60}\left[V\left(S43\right)-V\left(S36\right)\right]\\ +\frac{1}{60}\left[V\left(S44\right)-V\left(S13\right)\right]+\frac{1}{60}\left[V\left(S46\right)-V\left(S11\right)\right]+\frac{1}{60}\left[V\left(S47\right)-V\left(S37\right)\right]+\frac{1}{60}\left[V\left(S49\right)-V\left(S14\right)\right]\\ +\frac{1}{60}\left[V\left(S50\right)-V\left(S40\right)\right]+\frac{1}{60}\left[V\left(S51\right)-V\left(S12\right)\right]+\frac{1}{60}\left[V\left(S54\right)-V\left(S47\right)\right]+\frac{1}{60}\left[V\left(S55\right)-V\left(S33\right)\right]\\ +\frac{1}{60}\left[V\left(S56\right)-V\left(S45\right)\right]+\frac{1}{30}\left[V\left(S57\right)-V\left(S52\right)\right]+\frac{1}{30}\left[V\left(S58\right)-V\left(S15\right)\right]+\frac{1}{30}\left[V\left(S59\right)-\;V\left(S61\right)\right]\\ +\frac{1}{30}\left[V\left(S60\right)-\;V\left(S10\right)\right]+\frac{1}{30}\left[V\left(S62\right)-\;V\left(S60\right)\right]+\frac{1}{6}\left[V\left(S63\right)-\;V\left(S17\right)\right]. \end{array}$$

According to the formula, the final cost that Tianjin enterprises should bear is

(11) $$\begin{array}{c} Y_{i}\;\left(V\right)=\frac{1}{6}V\left(S16\right)+\frac{1}{30}\left[V\left(S18\right)-V\left(S16\right)\right]+\frac{1}{30}\left[V\left(S19\right)-V\left(S1\right)\right]+\frac{1}{30}\left[V\left(S20\right)-V\left(S2\right)\right]+\frac{1}{60}\left[V\left(S23\right)-V\left(S6\right)\right]\\ +\frac{1}{60}\left[V\left(S26\right)-V\left(S24\right)\right]+\frac{1}{60}\left[V\left(S27\right)-V\left(S22\right)\right]+\frac{1}{60}\left[V\left(S28\right)-V\left(S5\right)\right]+\frac{1}{30}\left[V\left(S30\right)-V\left(S23\right)\right]\\ +\frac{1}{30}\left[V\left(S33\right)-V\left(S10\right)\right]+\frac{1}{60}\left[V\left(S34\right)-V\left(S9\right)\right]+\frac{1}{60}\left.\left[V\left(S36\right)-V\left(S7\right)\right]\right]+\frac{1}{60}\left[V\left(S37\right)-V\left(S8\right)\right]\\ +\frac{1}{60}\left[V\left(S41\right)-V\left(S27\right)\right]+\frac{1}{60}\left[V\left(S43\right)-V\left(S14\right)\right]+\frac{1}{60}\left[V\left(S44\right)-V\left(S39\right)\right]+\frac{1}{60}\left[V\left(S46\right)-V\left(S12\right)\right]\\ +\frac{1}{60}\left[V\left(S46\right)-V\left(S42\right)\right]+\frac{1}{60}\left[V\left(S47\right)-V\left(S35\right)\right]+\frac{1}{60}\left[V\left(48\right)-V\left(S13\right)\right]+\frac{1}{60}\left[V\left(S51\right)-V\left(S11\right)\right]\\ +\frac{1}{60}\left[V\left(S52\right)-V\left(S38\right)\right]+\frac{1}{60}\left[V\left(S53\right)-V\left(S56\right)\right]+\frac{1}{60}\left[V\left(S55\right)-V\left(S50\right)\right]+\frac{1}{30}\left[V\left(S57\right)-V\left(S42\right)\right]\\ +\frac{1}{30}\left[V\left(S58\right)-V\left(S49\right)\right]+\frac{1}{30}\left[V\left(S59\right)-V\left(S15\right)\right]+\frac{1}{30}\left[V\left(S58\right)-V\left(S15\right)\right]+\frac{1}{30}\left[V\left(S60\right)-\;V\left(S62\right)\right]\\ +\frac{1}{30}\left[V\left(S62\right)-\;V\left(S60\right)\right]++\frac{1}{6}\left[V\left(S63\right)-\;V\left(S17\right)\right]. \end{array}$$

Therefore, through the above results, we can know that the total cost of governance is the cost borne by the three governments plus the cost borne by the enterprise is V (S15). In the air pollution control project, it is necessary to determine the total cost V (S15), the separate treatment cost V (S1) of the government in Beijing, and the cost V (S2) of the government alone to control air pollution. Therefore, through the above results, we can know that the total cost of governance is the cost borne by the three governments plus the cost borne by the enterprise is V (S15). In the air pollution control project, it is necessary to determine the total cost V (S15), the separate treatment cost V (S1) of the government in Beijing, and the cost V (S2) of the government alone to control air pollution. Hebei government alone treatment cost V (S3) and Hebei enterprise independent control cost V (S4), Tianjin government independent treatment cost V (S16), Tianjin enterprise independent treatment cost V (S17), by knowing the cost of the combination of the two of them, the cost of the combination of any three, the cost of the combination of any four, the combination of any five, and the cost of their joint governance, we can determine the respective costs borne by the government and enterprises in the treatment of air pollution in Beijing, Tianjin, and Hebei.

## 5. Example Analysis and Correction Based on Shapley Value

### 5.1. Numerical Calculation of Distribution Model

After collecting relevant data and sorting out the costs of air pollution control, we get the relevant costs for the treatment of air pollution in Beijing and Hebei. Taking Beijing and Hebei as examples, simplify the cost allocation model. Use A for Beijing Municipal Government, B for Beijing enterprises, C for Hebei provincial government, and D for Hebei enterprises, specific data as shown in Table 4.

According to the model established in the above section, the costs that Beijing municipal government, Beijing municipal enterprises, and Hebei provincial government should bear when establishing a cooperative alliance to control air pollution can be calculated. The specific results are shown in Table 5.

The sum of the data in the last row of the table can get the cost that Beijing government departments should bear in the joint governance of Beijing and Hebei. The final result is 229.167 billion Yuan, which is the optimal the cost. The specific results are shown in Table 6.

The sum of the data in the last row of the table can get the cost that Beijing enterprises should bear in the joint governance of Beijing and Hebei. The final result is 82.5 billion Yuan, which is the optimal cost. The specific results are shown in Table 7.

The sum of the data in the last row of the table can get the cost that the Hebei government should bear in the joint governance of Beijing and Hebei. The final result is 224.167 billion Yuan, which is the optimal cost. The specific results are shown in Table 8.

The sum of the data in the last row of the table can get the cost that enterprises in Hebei should bear in the joint governance of Beijing and Hebei region. The final result is 86.667 billion Yuan, which is the optimal cost.

### 5.2. Result Analysis

Based on the Shapley value method, when Beijing and Hebei implement joint governance, the total cost is 622.5 billion Yuan, which can effectively solve the cooperation needs of 620 billion Yuan. Meanwhile, Beijing municipal government departments bear 229.167 billion Yuan in the cooperative governance, Beijing enterprises bear 82.5 billion yuan of governance cost, the Hebei government bears 2,241 Yuan and 6.7 billion Yuan, and the cost borne by Hebei enterprises bear 86.667 billion yuan.

Because what is allocated as the cost, the Shapley value method is generally used for the distribution of income, so its assumption condition is generally positive; that is, the income obtained is positive; then on the contrary, the cost paid is negative; that is, A bears 229.167 billion yuan in cooperative governance, B bears 82.5 billion yuan, C bears 224.167 billion yuan, and D bears 86.667 billion yuan. According to the Shapley value allocation, the cooperation cost is shown in Table 9.

It can be seen from the above table that the cost borne by the cooperation is less than the cost generated by the individual governance, which also satisfies the individual rationality. At the same time, compared with the individual governance in each region, the cost borne by each stakeholder in the joint governance is significantly less than that borne by the individual governance. In the absence of relevant stakeholders, *V*(∅)=0 and *V*(*S*_1_ ∪ *S*_2_) ≥ *V*(*S*_1_)+*V*(*S*_2_) are satisfied.

To sum up, the cost obtained by using the Shapley value method is less than the cost of independent cooperation or independent governance, which can make the cost allocation more scientific, fair, and reasonable, reduce the risks borne by each stakeholder in participating in project governance, and promote the progress of the project governance. At the same time, in the actual situation, we must adjust the cost according to the actual situation and pay attention to risk control, to ensure the smooth completion of air pollution control.

### 5.3. Modifying the Model

Through the above analysis, the four benefit distribution factors, namely, cost bearing, risk bearing, contribution degree, and contract execution degree, should be considered. For convenience, the influential factors are set *T* = {*T*}, *T* = 1, 2, 3, and 4, respectively, representing these four factors. And in the cooperation mode set S of participants, the modification value of the influence factor on *t* cost allocation of the i^th^ participant is BIT. The specific results are shown in Table 10.

According to the above table, the following coefficient matrix B can be obtained:

(12) $$\begin{array}{c} B_{1}=\left[\begin{array}{c} b_{A1}\\ b_{A2}\\ b_{C1}\\ b_{D1}\\ b_{E1}\\ b_{F1} \end{array}\right],\\ B_{2}=\left[\begin{array}{c} b_{A2}\\ b_{B2}\\ b_{C2}\\ b_{D2}\\ b_{E2}\\ b_{F2} \end{array}\right],\\ B_{3}=\left[\begin{array}{c} b_{A3}\\ b_{B3}\\ b_{C3}\\ b_{D3}\\ b_{E3}\\ b_{F3} \end{array}\right],\\ B_{4}=\left[\begin{array}{c} b_{A4}\\ b_{B4}\\ b_{C4}\\ b_{D4}\\ b_{E4}\\ b_{F4} \end{array}\right]. \end{array}$$

If we arrange the matrix B, we get the matrix *B*′={*b*_*it*_′}_6×4_

In the process of atmospheric governance, several experts are needed to score the influencing factors. At this time, there will be a fractional coefficient matrix *A* = [A1, A2, A3, A4], and a new coefficient matrix *D* = *B*^*∗*^*A* = [*D*1, *D*2, *D*3, *D*4, *D*5, *D*6] can be obtained.

Therefore, after adjustment, the cost to be borne by each region is

(13) $$\begin{array}{c} Y_{i}^{\prime }\left(V\right)=\sum_{S_{i\;}\in S}W\left(\left|S\right|\right)\left[V\left(S\right)-V\left(S/i\right)\right]+D_{I}i\\ =1,2\ldots \text{n.} \end{array}$$

The adjusted Shapley value is closer to the reality, and more influential factors are considered so that the cost sharing is not only more objective but also to ensure the smooth implementation of the project so that the goal of atmospheric governance can be realized faster, and the cost distribution scheme is more fair, reasonable, and scientific.

## 6. Conclusion

This paper focuses on the issue across regional pollution control cost allocation. We established an air pollution control cost-sharing model based on the Shapley value and determined the core stakeholders to make the cost allocation more reasonable, scientific, and fair. The Shapley model reduces the charges of each stakeholder, disperses the risks of participants to a certain extent, and effectively ensures the smooth progress of the project. We found that the cost distribution model based on Shapley value can optimize the cost and maximize the social benefit. Because air pollution control needs a long process, the reduction of cost and risk can effectively ensure the completion of air pollution control, which plays an important role in promoting air pollution control.

The subsequent studies could consider factors such as risk, contribution rate, and the bearing capacity of each stakeholder. Determining the influencing factors according to the different situations of stakeholders can make the cost more reasonable and realistic. Besides, the governance in different regions is not the same. The prevention and control method based on the local conditions could make the cost allocation model more widely used, better solve the air pollution problem, and maximize social benefits.

## Figures and Tables

**Table 1:** Classification of stakeholders of air pollution control projects.

Stakeholders	Institutions	Mechanism classification basis
Core stakeholders	Local governments and enterprises in Beijing, Tianjin and Hebei	The indispensable participants of the air pollution control project have an inseparable interest with the control and cost sharing of the project
General stakeholders	Beijing-Tianjin-Hebei and surrounding areas' air pollution prevention and control collaborative group	Participants who are closely connected with air pollution control projects have a certain degree of project participation and bear certain risks
Marginal stakeholders	The central government	It has a little influence on air pollution control projects and does not directly contact each participant

**Table 2:** Making assumptions about the model.

A	B	C	D	E	F	Subset	Function	Number of participants
Participate in						*S*_1_	*V* (*S*_1_)	1
	Participate in					*S*_2_	*V* (*S*_2_)	1
		Participate in				*S*_3_	*V* (*S*_3_)	1
			Participate in			*S*_4_	*V* (*S*_4_)	1
Participate in	Participate in					*S*_5_	*V* (*S*_5_)	2
		Participate in	Participate in			*S*_6_	*V* (*S*_6_)	2
Participate in			Participate in			*S*_7_	*V* (*S*_7_)	2
	Participate in	Participate in				*S*_8_	*V* (*S*_8_)	2
Participate in		Participate in				*S*_9_	*V* (*S*_9_)	2
	Participate in		Participate in			*S*_10_	*V* (*S*_10_)	2
Participate in		Participate in	Participate in			*S*_11_	*V* (*S*_11_)	3
	Participate in	Participate in	Participate in			*S*_12_	*V* (*S*_12_)	3
Participate in	Participate in	Participate in				*S*_13_	*V* (*S*_13_)	3
Participate in	Participate in		Participate in			*S*_14_	*V* (*S*_14_)	3
Participate in	Participate in	Participate in	Participate in			*S*_15_	*V* (*S*_15_)	4
				Participate in		*S*_16_	*V* (*S*_16_)	1
					Participate in	*S*_17_	*V* (*S*_17_)	1
				Participate in	Participate in	*S*_18_	*V* (*S*_18_)	2
Participate in					Participate in	*S*_19_	*V* (*S*_19_)	2
	Participate in				Participate in	*S*_20_	*V* (*S*_20_)	2
	Participate in			Participate in		*S*_21_	*V* (*S*_21_)	2
			Participate in	Participate in		*S*_22_	*V* (*S*_22_)	2
Participate in				Participate in		*S*_23_	*V* (*S*_23_)	2
		Participate in		Participate in		*S*_24_	*V* (*S*_24_)	2
			Participate in		Participate in	*S*_25_	*V* (*S*_25_)	2
		Participate in			Participate in	*S*_26_	*V* (*S*_26_)	2
		Participate in	Participate in	Participate in		*S*_27_	*V* (*S*_27_)	3
		Participate in	Participate in		Participate in	*S*_28_	*V* (*S*_28_)	3
		Participate in		Participate in	Participate in	*S*_29_	*V* (*S*_29_)	3
			Participate in	Participate in	Participate in	*S*_30_	*V* (*S*_30_)	3
Participate in	Participate in			Participate in		*S*_31_	*V* (*S*_31_)	3
Participate in	Participate in				Participate in	*S*_32_	*V* (*S*_32_)	3
Participate in				Participate in	Participate in	*S*_33_	*V* (*S*_33_)	3
	Participate in			Participate in	Participate in	*S*_34_	*V* (*S*_34_)	3
Participate in		Participate in		Participate in		*S*_35_	*V* (*S*_35_)	3
	Participate in		Participate in		Participate in	*S*_36_	*V* (*S*_36_)	3
Participate in		Participate in			Participate in	*S*_37_	*V* (*S*_37_)	3
Participate in			Participate in	Participate in		*S*_38_	*V* (*S*_38_)	3
	Participate in	Participate in		Participate in		*S*_39_	*V* (*S*_39_)	3
Participate in			Participate in		Participate in	*S*_40_	*V* (*S*_40_)	3
	Participate in	Participate in			Participate in	*S*_41_	*V* (*S*_41_)	3
	Participate in		Participate in	Participate in		*S*_42_	*V* (*S*_42_)	3
Participate in	Participate in			Participate in	Participate in	*S*_43_	*V* (*S*_43_)	4
		Participate in	Participate in	Participate in	Participate in	*S*_44_	*V* (*S*_44_)	4
Participate in	Participate in		Participate in		Participate in	*S*_45_	*V* (*S*_45_)	4
	Participate in	Participate in		Participate in	Participate in	*S*_46_	*V* (*S*_46_)	4
	Participate in	Participate in	Participate in		Participate in	*S*_47_	*V* (*S*_47_)	4
	Participate in		Participate in	Participate in	Participate in	*S*_48_	*V* (*S*_48_)	4
Participate in	Participate in	Participate in		Participate in		*S*_49_	*V* (*S*_49_)	4
Participate in		Participate in	Participate in	Participate in		*S*_50_	*V* (*S*_50_)	4
Participate in		Participate in		Participate in	Participate in	*S*_51_	*V* (*S*_51_)	4
Participate in	Participate in	Participate in			Participate in	*S*_52_	*V* (*S*_52_)	4
Participate in		Participate in	Participate in		Participate in	*S*_53_	*V* (*S*_53_)	4
Participate in	Participate in		Participate in	Participate in		*S*_54_	*V* (*S*_54_)	4
Participate in			Participate in	Participate in	Participate in	*S*_55_	*V* (*S*_55_)	4
	Participate in	Participate in	Participate in	Participate in		*S*_56_	*V* (*S*_56_)	4
	Participate in	Participate in	Participate in	Participate in	Participate in	*S*_57_	*V* (*S*_57_)	5
Participate in		Participate in	Participate in	Participate in	Participate in	*S*_58_	*V* (*S*_58_)	5
Participate in	Participate in		Participate in	Participate in	Participate in	*S*_59_	*V* (*S*_59_)	5
Participate in	Participate in	Participate in		Participate in	Participate in	*S*_60_	*V* (*S*_60_)	5
Participate in	Participate in	Participate in	Participate in		Participate in	*S*_61_	*V* (*S*_61_)	5
Participate in	Participate in	Participate in	Participate in	Participate in		*S*_62_	*V* (*S*_62_)	5
Participate in	Participate in	Participate in	Participate in	Participate in	Participate in	*S*_63_	*V* (*S*_63_)	6

**Table 3:** Expenses borne by Beijing government departments in air pollution control projects.

A subset of S	*V*(*S*)	*V*(*S*\*i*)	[V(S) − V(*S*/*i*)]	W(|S|)	*W*(|*S*|)[*V*(*S*) − *V*(*S*/*i*)]
*S*1	*V*(*S*1)	0	*V*(*S*1)	1\6	1/46*V*(*S*1)
*S*5	*V*(*S*5)	*V*(*S*2)	*V*(*S*5) − *V*(*S*2)	1\30	1/30[*V*(*S*5) − *V*(*S*2)]
*S*7	*V*(*S*7)	*V*(*S*4)	*V*(*S*7) − *V*(*S*4)	1\30	1/30[*V*(*S*7) − *V*(*S*4)]
*S*9	*V*(*S*9)	*V*(*S*3)	*V*(*S*9) − *V*(*S*3)	1\30	1/30[*V*(*S*9) − *V*(*S*3)]
*S*11	*V*(*S*11)	*V*(*S*6)	*V*(*S*11) − *V*(*S*6)	1\60	1/60[*V*(*S*11) − *V*(*S*6)]
*S*13	*V*(*S*13)	*V*(*S*8)	*V*(*S*13) − *V*(*S*8)	1\60	1/60[*V*(*S*13) − *V*(*S*8)]
*S*14	*V*(*S*14)	*V*(*S*10)	*V*(*S*14) − *V*(*S*10)	1\60	1/60[*V*(*S*14) − *V*(*S*10)]
*S*15	*V*(*S*15)	*V*(*S*12)	*V*(*S*15) − *V*(*S*12)	1\60	1/60[*V*(*S*15) − *V*(*S*12)]
*S*19	*V*(*S*19)	*V*(*S*17)	*V*(*S*19) − *V*(*S*17)	1\30	1\30[*V*(*S*19) − *V*(*S*17)]
*S*23	*V*(*S*23)	*V*(*S*16)	*V*(*S*23) − *V*(*S*16)	1\30	1\30[*V*(*S*23) − *V*(*S*16)]
*S*31	*V*(*S*31)	*V*(*S*21)	*V*(*S*31) − *V*(*S*21)	1\60	1\60[*V*(*S*31) − *V*(*S*21)]
*S*32	*V*(*S*32)	*V*(*S*20)	*V*(*S*32) − *V*(*S*20)	1\60	1\60[*V*(*S*32) − *V*(*S*20)]
*S*33	*V*(*S*33)	*V*(*S*18)	*V*(*S*33) − *V*(*S*18)	1\60	1\60[*V*(*S*33) − *V*(*S*18)]
*S*35	*V*(*S*35)	*V*(*S*24)	*V*(*S*35) − *V*(*S*24)	1\60	1\60[*V*(*S*35) − *V*(*S*24)]
*S*37	*V*(*S*37)	*V*(*S*26)	*V*(*S*37) − *V*(*S*26)	1\60	1\60[*V*(*S*37) − *V*(*S*26)]
*S*38	*V*(*S*38)	*V*(*S*22)	*V*(*S*38) − *V*(*S*22)	1\60	1\60[*V*(*S*38) − *V*(*S*22)]
*S*40	*V*(*S*40)	*V*(*S*25)	*V*(*S*40) − *V*(*S*25)	1\60	1\60[*V*(*S*40) − *V*(*S*25)]
*S*43	*V*(*S*43)	*V*(*S*34)	*V*(*S*43) − *V*(*S*34)	1\60	1\60[*V*(*S*43) − *V*(*S*34)]
*S*45	*V*(*S*45)	*V*(*S*36)	*V*(*S*45) − *V*(*S*36)	1\60	1\60[*V*(*S*45) − *V*(*S*36)]
*S*49	*V*(*S*49)	*V*(*S*39)	*V*(*S*49) − *V*(*S*39)	1\60	1\60[*V*(*S*49) − *V*(*S*39)]
*S*50	*V*(*S*50)	*V*(*S*27)	*V*(*S*50) − *V*(*S*27)	1\60	1\60[*V*(*S*50) − *V*(*S*27)]
*S*51	*V*(*S*51)	*V*(*S*29)	*V*(*S*51) − *V*(*S*29)	1\60	1\60[*V*(*S*51) − *V*(*S*29)]
*S*52	*V*(*S*52)	*V*(*S*41)	*V*(*S*52) − *V*(*S*41)	1\60	1\60[*V*(*S*52) − *V*(*S*41)]
*S*53	*V*(*S*53)	*V*(*S*28)	*V*(*S*53) − *V*(*S*28)	1\60	1\60[*V*(*S*53) − *V*(*S*28)]
*S*54	*V*(*S*54)	*V*(*S*42)	*V*(*S*54) − *V*(*S*42)	1\60	1\60[*V*(*S*54) − *V*(*S*42)]
*S*55	*V*(*S*55)	*V*(*S*30)	*V*(*S*55) − *V*(*S*30)	1\60	1\60[*V*(*S*55) − *V*(*S*30)]
*S*58	*V*(*S*58)	*V*(*S*44)	*V*(*S*58) − *V*(*S*44)	1\30	1\30[*V*(*S*58) − *V*(*S*44)]
*S*59	*V*(*S*59)	*V*(*S*48)	*V*(*S*59) − *V*(*S*48)	1\30	1\30[*V*(*S*59) − *V*(*S*48)]
*S*60	*V*(*S*60)	*V*(*S*46)	*V*(*S*60) − *V*(*S*46)	1\30	1\30[*V*(*S*60) − *V*(*S*46)]
*S*61	*V*(*S*61)	*V*(*S*47)	*V*(*S*61) − *V*(*S*47)	1\30	1\30[*V*(*S*61) − *V*(*S*47)]
*S*62	*V*(*S*62)	*V*(*S*56)	*V*(*S*62) − *V*(*S*56)	1\30	1\30[*V*(*S*62) − *V*(*S*56)]
*S*63	*V*(*S*63)	*V*(*S*57)	*V*(*S*63) − *V*(*S*57)	1\6	1\6[*V*(*S*63) − *V*(*S*57)]

**Table 4:** Calculation of air pollution control costs (unit: 100 million Yuan).

Participants	Overhead expenses
A	7600
B	3200
C	7400
D	3000
A, B	7300
C, D	7200
A, D	7100
B, C	7050
A, C	7000
B, D	7150
A, C, D	6900
B, C, D	6800
A, B, C	6500
A, B, D	6700
A, B, C, D	6200

**Table 5:** Expenses borne by Beijing Government departments in air pollution control projects (unit: 100 million Yuan).

A subset of *S*	*V*(*S*)	*V*(*S*/*i*)	[V(S) − V(*S*/*i*)]	W(|S|)	W(|S|)[V(S) − V(*S*/*i*)]
*S*1	7600	0	7600	1/4	1900.00
*S*5	7300	3200	4100	1/12	341.67
*S*7	7100	3000	4100	1/12	341.67
*S*9	7000	7400	−400	1/12	−33.33
*S*11	6900	7200	−300	1/12	−25.00
*S*13	6500	7050	−550	1/12	−45.83
*S*14	6700	7150	−450	1/12	−37.50
*S*15	6200	6800	−600	1/4	−150.00

**Table 6:** Expenses borne by Beijing Enterprises in air pollution control projects. (unit: 100 million Yuan).

A subset of *S*	*V*(*S*)	V(*S*/*i*)	[V(S) − V(*S*/*i*)]	W(|S|)	W(|S|)[V(S) − V(*S*/*i*)]
*S*2	3200	0	3200	1/4	800.00
*S*6	7300	7800	−500	1/12	−41.67
*S*7	7100	7400	−300	1/12	−25.00
*S*10	7150	3000	4150	1/12	345.83
*S*11	6900	7200	−300	1/12	−25.00
*S*12	6800	7000	−200	1/12	−16.67
*S*14	6700	7150	−450	1/12	−37.50
*S*15	6200	6900	−700	1/4	−175.00

**Table 7:** Expenses borne by the Hebei Government in air pollution control projects. (unit: 100 million Yuan).

A subset of *S*	*V*(*S*)	*V*(*S*/*i*)	[V(S) − V(*S*/*i*)]	W(|S|)	W(|S|)[V(S) − V(*S*/*i*)]
*S*3	7400	0	7400	1/4	1850.00
*S*6	7200	3000	4200	1/12	350.00
*S*8	7050	3200	3850	1/12	320.83
*S*9	7000	7600	−600	1/12	−50.00
*S*11	6900	7100	−200	1/12	−16.67
*S*12	6800	7050	−250	1/12	−20.83
*S*13	6500	7300	−800	1/12	−66.67
*S*15	6200	6700	−500	1/4	−125.00

**Table 8:** Expenses borne by Hebei Enterprises in air pollution control projects (unit: 100 million Yuan).

A subset of S	*V*(*S*)	*V*(*S*/*i*)	[V(S) − V(*S*/*i*)]	W(|S|)	W(|S|)[V(S) − V(*S*/*i*)]
*S*4	3000	0	3000	1/4	750.00
*S*6	7200	7400	−200	1/12	−16.67
*S*7	7100	7600	−500	1/12	−41.67
*S*10	7150	3200	3950	1/12	329.17
*S*11	6900	7000	−100	1/12	−8.33
*S*12	6800	7050	−250	1/12	−20.83
*S*14	6700	7300	−600	1/12	−50.00
*S*15	6200	6500	−300	1/4	−75.00

**Table 9:** Cost of air pollution control (unit: 100 million Yuan).

Participants	Original governance cost	Cost based on Shapley value
A	−7600	−2291.67
B	−3200	−825.00
C	−7400	−2241.67
D	−3000	−866.67
A, B	−7300	−3116.67
C, D	−7200	−3108.33
A, D	−7100	−3158.33
B, C	−7050	−3066.67
A, C	−7000	−4533.33
B, D	−7150	−1691.67
A, C, D	−6900	−5400.00
B, C, D	−6800	−3933.33
A, B, C	−6500	−5358.33
A, B, D	−6700	−5400.00

**Table 10:** Correction coefficient table.

	1. (the expenses)	2. (risk taking)	3. (contribution)	4. (Degree of contract execution)
A	bA1	bA2	bA3	bA4
B	bB1	bB2	bB3	bB4
C	bC1	bC2	bC3	bC4
D	bD1	bD2	bD3	bD4
E	bE1	bE2	bE3	bE4
F	bF1	bF2	bF3	bF4

## Data Availability

The data of this project were obtained through the investigation of “National Joint Research Center for Air Pollution Prevention and Control Project Topic: Regional Dynamic and High Spatial-Temporal Resolution Air Pollution Source Emission Inventory.”

## References

[1] Aguilera R., Corringham T., Gershunov A., Leibel S., Benmarhnia T. (2021). Fine particles in wildfire smoke and pediatric respiratory health in California. *Pediatrics*.

[2] Meng J., Wang M., Xuekelaiti X. (2021). Characteristics of air pollution and environmental economic efficiency in Beijing-Tianjin-Hebei and surrounding areas. *Arabian Journal of Geosciences*.

[3] Xin L. A., Hz B., Tao X. C. (2021). Consumption-based PM 2.5 -related premature mortality in the Beijing-Tianjin-Hebei region. *The Science of the Total Environment*.

[4] Jiao Y., Su M., Ji C., Yang S. (2021). How to design fully cooperative policies to abate transboundary air pollution between two highly asymmetric regions: an abnormal incrementalism analysis. *Journal of Cleaner Production*.

[5] Yan H. A., Xn B., Jw C. (2021). Impacts of haze pollution on China’s tourism industry: a system of economic loss analysis. *Journal of Environmental Management*.

[6] Zhao C., Deng M., Cao X. (2021). Does haze pollution damage urban innovation? Empirical evidence from China. *Environmental Science and Pollution Research*.

[7] Yang Z., Jing S., Yu L. (2018). Atmospheric environment vulnerability cause analysis for the beijing-tianjin-hebei metropolitan region. *International Journal of Environmental Research and Public Health*.

[8] Liang L., Wang Z. (2021). Control models and spatiotemporal characteristics of air pollution in the rapidly developing urban agglomerations. *International Journal of Environmental Research and Public Health*.

[9] Sun L., Du J., Li Y. (2021). A new method for dividing the scopes and priorities of air pollution control based on environmental justice. *Environmental Science and Pollution Research*.

[10] Piersanti A., D’Elia I., Gualtieri M. (2021). The Italian national air pollution control Programme: air quality, health impact and cost assessment. *Atmosphere*.

[11] Ikeuchi H., Murakami M., Watanabe S. (2015). Scavenging of PM2.5 by precipitation and the effects of precipitation pattern changes on health risks related to PM2.5 in Tokyo, Japan. *Water Science and Technology*.

[12] Schwartz J., Laden F., Zanobetti A. (2002). The concentration-response relation between PM(2.5) and daily deaths. *Environmental Health Perspectives*.

[13] Gulia S., Tiwari R., Mendiratta S., Kaur S., Goyal S. K., Kumar R. (2020). Review of scientific technology-based solutions for vehicular pollution control. *Clean Technologies and Environmental Policy*.

[14] Elżbieta S. T. (2021). Anti-smog building and civil engineering structures. *Processes*.

[15] Wr A., Ss B., Hs A. (2021). A review on the deteriorating situation of smog and its preventive measures in Pakistan. *Journal Of Cleaner Production*.

[16] Zhao Q., Yuan C. H. (2020). Did haze pollution harm the quality of economic development?-an empirical study based on China’s PM2.5 concentrations. *Sustainability*.

[17] Wang Z., Hu W., Niu H. (2020). Variations in physicochemical properties of airborne particles during a heavy haze-to-dust episode in Beijing. *The Science of the Total Environment*.

[18] Gen M., Zhou L., Zhang R., Chan C. K. (2021). Concluding remarks: faraday Discussion on air quality in megacities. *Faraday Discussions*.

[19] Zhang X., Cai X. H., Chai F. H. (2006). Structures and characteristics of the atmospheric boundary layer over Beijing area in autumn. *Acta Scientiarum Nauralium Universitaties Pekinensis*.

[20] Ren X., Qu R., Liu S. (2020). Synthesis of zeolites from coal fly ash for removal of harmful gaseous pollutants: a review. *Aerosol and Air Quality Research*.

[21] Wang Q., Yuan B. (2018). Air pollution control intensity and ecological total-factor energy efficiency: the moderating effect of ownership structure. *Journal of Cleaner Production*.

[22] Kim B., Yoon E. J., Kim S., Lee D. K. (2020). The effects of risk perceptions related to particulate matter on outdoor activity satisfaction in South Korea. *International Journal of Environmental Research and Public Health*.

[23] Zhao L., Xue J., Gao H. O., Li C., Huang R. (2014). A model for interprovincial air pollution control based on futures prices. *Journal of the Air & Waste Management Association*.

[24] Gao Y., Guo X., Ji H., Li C. (2016). Potential threat of heavy metals and PAHs in PM2.5 in different urban functional areas of Beijing. *Atmospheric Research*.

[25] Colini-Baldeschi R., Scarsini M., Vaccari S. (2018). Variance allocation and shapley value. *Methodology and Computing in Applied Probability*.

[26] Guo B., Hao S., Cao G., Cao H. (2021). Profit distribution of liner alliance based on shapley value. *Journal of Intelligent and Fuzzy Systems*.

[27] Wang L., Li Y., Wang Y. (2021). Compensation benefits allocation and stability evaluation of cascade hydropower stations based on Variation Coefficient-Shapley Value Method. *Journal of Hydrology*.

[28] Garratt R. (2019). An application of shapley value cost allocation to liquidity savings mechanisms. *Staff Working Papers*.

[29] Aas K., Jullum M., Lland A. (2019). Explaining individual predictions when features are dependent: more accurate approximations to Shapley values. *Artificial Intelligence*.

[30] van den Brink R., Pintér M. (2015). On axiomatizations of the shapley value for assignment games. *Journal of Mathematical Economics*.

[31] Kim S. (2016). Asymptotic shapley value based resource allocation scheme for IoT services. *Computer Networks*.

[32] Liao Z., Zhu X., Shi J. (2014). Case study on initial allocation of Shanghai carbon emission trading based on Shapley value. *Journal of Cleaner Production*.

[33] Meng F.-Y., Zhang Q. (2010). The Shapley function for fuzzy cooperative games with multilinear extension form. *Applied Mathematics Letters*.

[34] Wei G., Zhang N. (2014). A multiple criteria hesitant fuzzy decision making with Shapley value-based VIKOR method. *Journal of Intelligent and Fuzzy Systems*.

